The article "Removing blurring for better understanding the main challenges facing digital entrepreneurs in the digital era: An empirical investigation study from emerging country" was retracted in 2024. Reasons: duplicate publication; overlap with earlier publications.

# Removing blurring for better understanding the main challenges facing digital entrepreneurs in the digital era: An empirical investigation study from emerging country

**DOI:** 10.1016/j.heliyon.2024.e25150

**Published:** 2024-01-28

**Authors:** Moh'd Anwer AL-Shboul

**Affiliations:** Business Administration Department, King Talal School of Business Technology, Princess Sumaya University for Technology (PSUT), P.O. Box 1438 Al-Jubaiha, Amman, Jordan

**Keywords:** Digital entrepreneurs, Entrepreneurship challenges, Early startups, Artificial intelligence, Developing countries

## Abstract

The purpose of this study is to examine the main challenges that these entrepreneurs in developing nations confront. This study utilizes a digital startup database maintained by the Ministry of Digital Economy and Entrepreneurship (MoDEE) in Jordan and conducts semi-structured interviews with a random selection of 85 early-stage digital entrepreneurs. In order to understand the cognitive and psychological characteristics of digital entrepreneurs and their motives for entering the field, this study draws on the theory of planned behavior. Using NVivo 20, a theme analysis is carried out. Based on the interviews conducted, the top industries among the startups that were looked at were big data and business analytics, internet-of-things (IoT), cybersecurity (CT) technology, food service and agri-tech, warehouse automation (WA) and elastic logistics (ELs), conversional artificial intelligence (CAI), financial technology (FinTech), and block chain technology (BCT). 42.5 % of the target population is represented by the large sample size that was used. These obstacles could include long-term funding, a dearth of one-on-one coaching and guidance, unforeseen risks or setbacks, and financial constraints. The study's conclusions may provide policymakers with a tactical manual for removing the main barriers that emerging digital entrepreneurs and their firms must overcome.

## 1 Introduction

Using the Schumpeter effect in developing nations [1], entrepreneurship is a way to fight unemployment and poverty [2]. Jordan's unemployment rate as of the third quarter of 2022 was above 23 % [3], a notable rise from 15.27 % in 2016 [4]. Elevated jobless rates have an adverse influence on the establishment of new enterprises, with the consequences differing according to the industry, region, and other variables [5], and [6]. found a negative relationship between unemployment and entrepreneurship [7]. People who are trying to break free from the grip of unemployment frequently turn to entrepreneurship as a workable alternative. However, there are many obstacles in the way of this voyage [8]. The demand for digital products increased because of the COVID-19 pandemic's instigation of a digital revolution [9]. This circumstance expedited the introduction of Digital Entrepreneurs (DEs) into the market by presenting new opportunities [10]. Because of these special chances and competitive advantages the epidemic has given them, DEs are different from typical entrepreneurs. Nevertheless, these prospects have also brought new risks and challenges for DEs, which could have an impact on their ability to succeed as a business. These include shifts in the market, problems with infrastructure and technical preparedness, and worries about financial support [11], and [12].

In Jordan, obtaining funding, paying hefty taxes, and dealing with frequent rule and regulation changes are major obstacles to entrepreneurial endeavors [13]. The government and allied sectors urgently need to expedite technology adoption and simplify procedures for entrepreneurs, even in spite of a forward-looking goal for digital transformation that extends to 2025 [14]. Entrepreneurs have also discovered other administrative and cultural barriers, motivated by both necessity and opportunity [15].

This study focuses on the challenges faced by early-stage DEs (those whose companies are under a year old) in Jordan due to the paucity of research on the issues facing DEs in developing countries, and particularly in Jordan. The following questions are the focus of this research and are meant to help us better understand them:

1. What are the main difficulties encountered by early-stage DEs in Jordan?
2. What suggestions can be proposed to overcome these difficulties?

To tackle the previously indicated inquiries, a qualitative approach employing thematic analysis via semi-structured interviews is employed. The study involved 85 early-stage Digital Entrepreneurs (DEs) who were chosen at random. They worked in a variety of industries, such as big data and business analytics, food service and agriculture technology (AgriTech), last-mile delivery technology (LMDT), cybersecurity technology (CT), conversional artificial intelligence (AI), warehouse automation (WA), education technology (EDTech), leisure and entertainment, financial technology (FinTech), wearable technology (WT), cloud-based SaaS solutions, digital healthcare technology, internet-of-things (IoTs), block chain technology (BCT), supply chain and elastic logistics, online retail (OR), and virtual reality (VR).

This study focuses on the most significant barriers and difficulties that Jordanian digital entrepreneurs face, particularly given that their nation is still developing. As a result, as some of the following points demonstrate, this study aims to close some research gaps in the area of digital entrepreneurs:

➢ After reviewing the literature on entrepreneurs in general, it was discovered that, because Jordan is a developing nation, any one-model framework did not cover the primary difficulties and barriers faced by digital entrepreneurs there.
➢ There were relatively few studies undertaken in developing countries compared to the large number of studies conducted in wealthy countries on the same subject matter in the past.

The purpose of this study is to provide a thorough, quantitative, and descriptive evaluation that takes into account the unique characteristics of entrepreneurs. These characteristics include their knowledge of and comfort with information and communications technology (ICT), their comprehension of technology, their resource-based skills, their financial situation, and their perspectives and attitudes on society and technology. Additionally, the study aims to provide in-depth analyses of the surrounding environment. This covers aspects such as government policies, market difficulties and possibilities for digital entrepreneurship, societal and industrial e-readiness, societal trust levels, and the state of the financial market [16].

## 2 Theoretical background and literature review

### 2.1 Digital entrepreneurship

Many views of entrepreneurship are available in the literature [17]. [18] defined it as the search for new opportunities. It frequently has to do with the creation of a new organization or the restructuring of an old one [19]. According to Drucker's (1985) connection between entrepreneurship and innovation, the former entails creative actions that optimize the use of available resources in order to create wealth. Other studies link entrepreneurship to opportunity detection and preemptive measures [20,21], and [22].

By the middle of the seventeenth century, the word “entrepreneur” had its start. Cantillon (1755) described an entrepreneur as a person who buys products with the intention of selling them later for a specific purpose [23]. defined an entrepreneur as a person who uses scarce resources to further their own interests [24]. indicated that an entrepreneur is versatile enough to perform in varied situations and is distinguished by innovativeness and risk-taking inclination. An entrepreneur's path usually begins with problem identification and transformation into concrete opportunity [25].

The idea of a “entrepreneur” has evolved over time, and studies have been conducted on the characteristics of prosperous businesspeople. A distinctive and diverse set of attributes, including patience, optimism, and outstanding communication abilities, make an entrepreneur stand out [22,26], and [19]. Entrepreneurs are charismatic people who captivate others when it comes to leadership and team building [27].

Different types of entrepreneurs exist [28], as well as [29]. [30] classified business owners according to their character traits [31]. divided them into two groups: operators and visionaries. Six essential processes are typically followed by operators who have not yet launched their product or have not scaled their companies to a suitable degree: selection, execution, assignment, allocation, monitoring, and modification. On the other hand, visionaries typically focus on determining the issue and developing a long-term solution strategy. They concentrate on laying out the essential procedures and then creating plans for managing human resources. Learning, establishing goals, creating, motivating, and keeping an eye on things are common tasks for visionaries. No matter how they are classified or what kind of firm they run, entrepreneurs usually want to introduce novel answers to problems that affect people. [32], and [33].

“Push and pull” entrepreneurship has been discussed in previous research under a theoretical framework [6 [34], and [35]. As per reference [36], “push” entrepreneurship is commonly associated with elements that motivate an individual to initiate entrepreneurial endeavors. This frequently involves them being dissatisfied with their current job, which motivates them to look for self-employment. People typically become involved in this type of entrepreneurship as a result of unfavorable situations [37]. On the other hand, “pull” entrepreneurship is associated with initiative, financial rewards, and a desire for success. This kind involves the entrepreneur proactively recognizing an issue and looking for fixes [36]. Different countries and generations have different motivating elements for these two types of entrepreneurship [38], and [35].

Technology is included into a digital startup's first business strategy in at least one significant way [39]. Due of their strong connections to information and communication technology (ICT) [40,41], and other related fields, digital entrepreneurs (DEs) straddle many business classification groups [42]. [43] refer to business prospects that use technology to solve specific problems as digital entrepreneurship. Digital entrepreneurship is a novel phenomena wherein digital technologies, processes, and infrastructure come together to exploit opportunities and handle developing issues [44,45], and [46].

The connection between digital transformation and digital entrepreneurship has been studied in recent years [25,47,48,49,9], and [45]. This relationship connects with the concepts of supply and demand. The supply side is made up of people who can operate as entrepreneurs in a variety of environments. Conversely, the chances for employment that entrepreneurs can fill are represented by the demand side [50]. Digital transformation initiatives have the potential to benefit entrepreneurs [[51], [52]], and [53].

The COVID-19 epidemic has reshaped the ecosystem in terms of potential exploitation and mental processes, creating a new route for entrepreneurship [54]. Studies examining the patterns in digital transformation and innovation have proliferated recently [55].

### 2.2 Digital entrepreneurship in Jordan

In order to understand the cognitive and psychological components of DEs and their reasons for pursuing digital entrepreneurship, this research draws on the theory of planned behavior [56]. Furthermore, this theory is frequently utilized to clarify the components and mechanisms that lead to the adoption of entrepreneurship and the ambition to pursue entrepreneurship. It considers the variables affecting people's intentions, which in turn control the outward actions taken in relation to an activity. As a result, the theory helps clarify how the perception and cognitive processes of the entrepreneurs, when influenced by external variables, may affect their intention to engage in digital entrepreneurship. This study is significant because it focuses on Jordan, a particular developing nation, and examines its particular difficulties in the area of digital entrepreneurship—a subject not well explored in prior studies. This study is important because it examines the difficulties that digital entrepreneurs face not only in developing nations generally but also in Jordan specifically, in taking into account infrastructure, financial and legal requirements, and other factors. The study also recognizes the impact of geographic and cultural elements, which have a considerable impact on the characteristics of concepts, services, and goods [57]. While comparable studies usually use quantitative approaches, this research adds to the body of knowledge by employing a semi-structured questionnaire and a qualitative approach. since of this, the qualitative technique is considered valuable since it can reveal new information that a quantitative method could miss [58], and [59].

Middle Eastern nations, like Jordan, which is a developing country in the region, are concentrating on encouraging an entrepreneurial culture in order to tackle the high rates of youth unemployment [60]. Support for relevant rules and regulations has grown ever since entrepreneurship started to gain traction in Jordan [61].

Jordan has made noteworthy progress in the Global Entrepreneurship Index, moving up from 72nd place in 2014 to 49th place in 2018, as part of the push to encourage entrepreneurial activity to produce employment and cut unemployment. When compared to economically prosperous neighboring nations like Saudi Arabia and the United Arab Emirates (UAE), Jordanian entrepreneurs have exhibited remarkable performance in areas such as startup skills, product innovation, and networking [62], as indicated in Fig. 1.

**Fig. 1:** Comparing Jordan's position in the 14th Global Entrepreneurship Index with respect to neighboring countries (preference through higher scores). (Source: MoDEE, 2022).

Twenty-seven firms from Jordan participated in the World Economic Forum in 2019—an occasion that gathered the top 200 startups in the Arab world [63]. Jordan replaced the Ministry of Information and Communications Technology and the Ministry of Digital Economy and Entrepreneurship (MoDEE) as part of its commitment to improve the business climate and hasten digitalization. This action, which emphasized the critical role that technology plays in corporate operations, was intended to support entrepreneurial endeavors by boosting startups, encouraging networking and collaboration, and improving funding access [64].

Small and Medium Enterprises (SMEs) play a crucial part in Jordan's economy, as evidenced by the fact that they account for an astounding 96 % of the country's GDP. Recognizing this, the government has emphasized on growing this sector to alleviate job difficulties [65]. Working together, decision-makers hope to remove barriers and preserve a climate that supports the dreams of young people who want to become entrepreneurs. These days, Jordan has more than twenty different organizations—private, public, and nonprofit—that provide a wide range of activities for business owners. iPark is committed to administering intellectual property rights registration, providing chances for incubation, and accelerating the growth of companies. The Queen Rania Center for Entrepreneurship (QRCE) offers a variety of services in collaboration with other organizations to support digital entrepreneurship. The main objectives of QRCE are to finance entrepreneurial endeavors, promote networking, and increase awareness. A private company called Oasis 500 provides early- and mid-stage businesses with funding, mentoring, and incubation; it often targets technology-related ventures [66], and [67].

During the COVID-19 epidemic, Jordan's unemployment rate increased, especially for young people, where it reached about 37 %. At the same time, fewer new businesses were established in the nation [68]. Fig. 2 shows Jordan's New Business Density (NBD) and the number of registered limited liability companies (LLCs) between 2010 and 2020.

**Fig. 2:** The number of registered firms with limited liability and the New Business Density during the years from 2010 to 2020 in the State of Jordan. (Source: The World Bank, 2022a).

According to Ref. [69], the number of recently registered corporations per 1000 people of working age (those who are fifteen to sixty-four years old) is the definition of the New Business Density (NBD).The NBD was about half of what it was in 2013 in 2020, a dramatic decline. In addition, between 2018 and 2020, Jordan had a decline in the quantity of newly formed Limited Liability Companies (LLCs). Jordan's economy and economic environment were severely impacted by the COVID-19 epidemic, but the nation's digital entrepreneurship scene continued to rise in the Middle East and North Africa (MENA) area. During this time, a number of Jordanian businesses were successful in raising venture financing [63].

Comparing digital entrepreneurship in developed and underdeveloped nations is crucial. Because they are e-readiness and have the infrastructure to support it, advanced nations, such as those in Europe and the Americas, have started to embrace digital entrepreneurship. The significant shift in global business brought about by ongoing technology transformations is further highlighted in the literature [70].

### 2.3 Challenges facing digital entrepreneurship

The majority of prior research suggests that the difficulties and impediments faced by digital entrepreneurs stem from the insufficient capital needed to launch entrepreneurial ventures and enterprises, particularly in developing nations with underdeveloped banking systems and weak economies. The founders also lack the credit history and collateral necessary to obtain conventional bank loans [71,26]. From this vantage point, the general lack of supply frequently restricts access to the cash required for the work of innovative digital initiatives, and the owners of these businesses are typically members of the financially insufficient classes. As a result, they turn to borrowing from outside parties, where the dangers are higher. This is just one of the difficulties and barriers that face digital entrepreneurs generally. Therefore, special financing institutions are formed to facilitate smooth borrowing operations and field teams are formed to meet with entrepreneurs in the field in order to identify the most important challenges facing their entrepreneurial projects and to build trust relationships for transactional relationships in order to address these sensitive issues and reduce the risks that digital entrepreneurs may face [72].

Due to their high unemployment rates, most developing countries' economies face numerous obstacles in their daily operations. These include the dearth of funding needed for digital entrepreneurship, as well as the difficulty of securing the funds needed to establish and implement these initiatives locally. A lack of funding, a subpar educational system, and strict regulatory frameworks are some of the issues facing digital entrepreneurship in developing countries generally, and Jordan specifically. Other barriers include social stigma and unfavorable attitudes toward the practice. The psychological components of entrepreneurship and the focus on other elements of the business environment are the two main schools of thought that are usually against digital entrepreneurship [53].

Macro environmental issues are worth taking into account because they can have an impact on digital entrepreneurship. Key impediments also include other variables that influence the macro-environment, such as the requirement for financial support, bureaucracy, an insufficient regulatory and facilitation system, an inadequate educational system, and a lack of training in digital entrepreneurship [18]. Specifically, instability in politics, corruption, inadequate infrastructure, education, and training, in addition to a lack of capital, are major hindrances to the success of digital entrepreneurs in developing countries. Since most digital entrepreneurs are unable to keep up proper credit records, adequate business strategies, and collateral, financial banks are reluctant to provide loan help to them. In addition, personality traits, educational standards, individual family unit structure, and present degrees of personal desire are considered to have the greatest effects on digital entrepreneurial start-up activities.

## 3 Methodology

### 3.1 Study roadmap

This study explores the challenges faced by digital entrepreneurs through the application of thematic analysis and a qualitative approach to data collection, as illustrated in Fig. 3's roadmap. This type of strategy, according to Ref. [73], includes any research that produces findings not found through statistical analysis or other quantitative techniques. The qualitative nature of the inquiry, which includes observing the person's life, experiences, and behavioral traits as well as social movements, cross-national relationships, sentiments, and feelings, serves to highlight the study. Additionally, it included social patterns, cultural characteristics, organizational sentiments, and cross-national interactions [74,75]. Therefore, the multidisciplinary nature of qualitative research facilitates a comprehensive knowledge of a particular event, and its specificity ensures that it invariably produces concrete results that are both thought-provoking and true to life. Furthermore, it incorporates an integration of multidisciplinary features that offer a deep understanding of a specific event as well as an assessment of the nature of the outcomes and the significance they provide in addition to the idea projection [76], and [77]. As a result, qualitative interviews are renowned for being successful in illuminating unique perspectives, histories, and points of view about a given topic [78]. Using case studies from start-ups in Jordan's environment as a developing nation through in-person semi-structured interviews, a qualitative approach was taken [79,80]. Case studies are thought to be an appropriate approach that can provide and gather rich data, gather and examine detailed information and understanding regarding the primary obstacles faced by digital entrepreneurs in the context of the digital era, and additionally identify contextual effects that align with our research objectives [81], and [78]. Prior to data collection in its final version, all questions were forwarded to six separate academic instructors and practitioners who work and specialize in this topic in order to achieve a high degree of validation, as advised by Ref. [23]. This ensured the content validity of all questions. Samples of the items and questions that were part of the chosen constructs, variables, and challenges during the semi-structured interview process are displayed in Table 1.

**Fig. 3:** Study's roadmap. (Source: Author's own work).

**Table 1:** Shows samples of items and questions included in the selected constructs/variables/challenges during the conducting semi-structured interviews (n = 85). (Source: Author's own work).

Construct/Challenge	Interviewers' Items/questions	Interviewees Answers	#. of shared and consistent answers of the Interviewees (n = 85)
*Challenge 1: Weakness in the funding required within fair, realistic conditions and criteria.*	Do you think the funds are enough to startup your business?	*Participant opinion: “The funding required varies depending on the scope of the idea and the necessary software and hardware. Additionally, it is essential to take into account the costs associated with marketing and operations*". *Manager opinion: “The Ministry of Digital Economy and Entrepreneurship provides the necessary IT infrastructure for entrepreneurs to facilitate communication processes internally and externally and provides the necessary financial support and financing for the success of their businesses and facilitates procedures"*	16
*Challenge 2: Weaknesses and failures in the face of unexpected risks*	Can you talk freely about the main weakness and unexpected risk that your startup faced before and during launching it?	*Participant opinion: “Risks are ever-present in various aspects, encompassing technical challenges, market uncertainties, financial risks, and geopolitical instabilities in the region".* *Manager opinion: “Any entrepreneurial idea within the scope of digital entrepreneurship, the element of risk in its application is present, but in different proportions commensurate with the size and type of the entrepreneurial idea presented in its chances of success".*	14
*Challenge 3: Weakness in providing the necessary advice and continuous guidance*	Tell me frankly; about if there are any weakness in providing the necessary advices and continuous guidance from Ministry of Digital Economy and Entrepreneurship in Jordan.	*Participant opinion: “At first glance, the university appears to be promoting the entrepreneurial culture through entrepreneurship centers and incubators. However, upon closer examination, it becomes apparent that digital entrepreneurs are left to face the challenges on their own".* *Manager opinion: “The ministry has a qualified staff to provide advice, guidance, and advice to digital entrepreneurs, as well as reduce the obstacles and challenges that they may face before and during the start-up company"*	13
*Challenge 4: Economic barriers and challenges*	Can you tell me frankly about if there is any economic barriers and challenges that faced your startup during and after launching your business?	*Participant opinion: “The operational expenses associated with advanced technology create challenges for DEs themselves and these challenges are ultimately passed on to customers".* *Manager opinion: “From the Ministry's point of view, technological and operational costs are among the most important challenges and economic obstacles for digital entrepreneurs".*	17
*Challenge 5: Challenges of intense competitive pressures locally, regionally, and globally*	Can you give me your opinion about the main challenges and intense competitive pressures locally, regionally, and globally that face your startup after lunching your business?	*Participant opinion: “It is challenging for me to compete with major website/app builders globally who leverage a multitude of ready-made templates and sometimes charge customers exclusively for hosting services. In contrast, I dedicate hours to programming, customization, and design".* *Manager opinion: “Most of the large-scale companies working in digital entrepreneurship and startups are modernizing their operational, administrative, and logistical systems and adopting the latest technological technologies to keep pace with the rapid developments to serve customers in a more distinctive way regionally and globally than companies with limited resources and capabilities in their scope of work and capabilities locally".*	14
*Challenge 6: Weakness providing and adopting a friendly environment and sustainability for entrepreneurs.*	Tell me freely about the main weakness of your startup as digital entrepreneur for providing and adopting a friendly environment and sustainability for offering products and services for your customers.	*Participant opinion: “We offer all necessary resources so that we can environmentally be friendly so that we can compete with other projects to obtain adequate support for our startup economically and morally by accelerating the economic measures supporting us and providing all the necessary sources for the success of our creative ideas and our applications on the ground for customers”.* *Manager opinion: “The Ministry provides adequate support of all kinds, whether material or moral green, as well as facilitation and speed in procedures for startups and digital entrepreneurs in providing everything necessary for the success of their entrepreneurial projects in a short time and become more sustainable with dynamic environments".*	11

### 3.2 Study sample and data collection

A sample of 85 digital entrepreneurs (DEs) were used in the study; they were chosen at random from the businesses Jordan database, which has 546 businesses overall, 200 of which are early-stage DEs (less than a year old). The Innovative Startups and SMEs Fund (ISSF) provides financing to the Information and Communications Technology Associations, which in turn operate the Startups Jordan database, which is hosted by the Ministry of Digital Economy and Entrepreneurship (MoDEE). Businesses Jordan acts as a conduit for relationships between investors, influential figures in the entrepreneurial space, and businesses. It gives vital details about every business, like its age and area of expertise. Furthermore, the platform creates opportunities for collaboration among entrepreneurs, with a particular focus on digital projects spanning various domains, including agriculture, food, education, finance, 3D printing, blockchain, Artificial Intelligence (AI), e-commerce, and other fields (Startups JO, 2022).

A combination of synchronous time communication and asynchronous place communication techniques, like phone calls and videoconferencing, were used to collect data. These techniques were selected due to their adaptability in contrast to synchronous time and location communication systems [82,83]. One of the founder members of each firm was interviewed in a semi-structured manner to allow for freedom in the questions asked and to enable the interviewees to freely share their comments [84]. To make sure that nothing was missed, thorough notes were made both during and just after the interviews. Prior to further processing and analysis, the interviewees were interviewed regarding the recorded notes to confirm the authenticity and correctness of the material.

Based on where they were physically located, the early DEs were divided into two groups: the first group operated out of independent incubators, while the second group was based out of entrepreneurship and innovation centers of Jordanian public and private institutions. Table 2 illustrates the differences in the industry, number of LLCs, and average interview duration for the 85 interviews.

**Table 2:** Evidence of data gathered. (Source: Author's own work).

Digital Startups Sector	(No. of Industries Interviewed, No. of LLC)	Average Interview Time (in min.)
**Big data & Business Analytics**	(6,2)	72
**Food Service &Agriculture Technology (AgriTech)**	(4, 2)	64
**Last-Mile Delivery Technology (LMDT)**	(3,1)	59
**Cybersecurity Technology (CT)**	(5,1)	61
**Conversional Artificial Intelligence (AI)**	(5, 2)	58
**Warehouse Automation (WA)**	(6, 2)	62
**Education Technology (EDTech)**	(4, 1)	48
**Leisure & Entertainment**	(6, 2)	68
**Financial Technology (FinTech)**	(6, 2)	42
**Wearable Technology (WT)**	(4, 1)	54
**Cloud-based SaaS Solutions**	(6, 1)	64
**Digital Healthcare Technology**	(4, 1)	46
**Internet-of-Things (IoTs)**	(4, 10)	60
**Block chain Technology (BCT)**	(5, 1)	38
**Supply Chain and Elastic Logistics**	(6, 1)	46
**Online Retail (OR)**	(7, 1)	52
**Virtual Reality (VR)**	(4,1)	42
Decision Maker in Ministry of Digital Economy and Entrepreneurship (MoDEE)	**(No. of Managers Interviewed, No. of LLC)**	**Average Interview Time (in min.)**
**Top manager/President-Vic President**	(3, 2)	72
**Chief executive manager-officer/director**	(6, 3)	54
**Senior manager**	(4, 1)	42
**First line manager**	(2, 2)	28

85 DEs made up the study's sample; 27 % were female and 73 % were male. The ages of the entrepreneurs varied, as Fig. 4 illustrates. Of them, 36 % were undergraduates, 41 % were between the ages of 26 and 35, and the remaining percentage was 36 years and above.

**Fig. 4:** Distribution of digital startups entrepreneurs by Age and Gender. (Source: Author's own work).

Based on where they operated the early digital entrepreneurs (DEs) were split into two groups: those operating from independent incubators and those functioning from entrepreneurship and innovation centers within Jordanian public and private universities. Table 2 shows that among the 85 interviews, the industry, quantity of Limited Liability Companies (LLCs), and average interview length differed.

Every startup that was looked at during the study period was under a year old. Of them, 42.4 % were registered, while the remaining 57.6 % were still in the process of registering or getting a business license. As shown in Fig. 5, the registered firms were divided into three main legal categories: corporation, Limited Liability Company (LLC), and sole proprietorship.

**Fig. 5:** The emerging digital entrepreneurship firms that were interviewed by legal type and their registration status as a startup business. (Source: Author's own work).

The participants work in a variety of industries, such as cybersecurity, e-commerce, data and AI, entertainment, health technology, and agriculture technology. When asked about their other sources of income, 38 % of the DEs said they worked as independent contractors, part-timers, or full-timers, while 62 % said their only sources of income are their family and their entrepreneurial endeavor.

### 3.3 Data analysis and interpretation

Thematic analysis, as suggested by Ref. [85], was used for this investigation. First, the interviews were transcribed, and care was taken to record all notes taken both during and after each interview. NVivo 20 was the main software utilized for the study, with Microsoft Word being used in conjunction with its comment capability. Certain codes were allocated to statements in NVivo; characteristics like color and frequency helped categorize these codes. The 85 interview codes were arranged in a methodical manner to enable the differentiation of data for every single interview. Ultimately, the nodes holding different codes were where the major themes came from. It is noteworthy that the study mostly focused on shared points among the interviewees, with limited verbatim usage.

## 4 Results and discussion

Risks for digital entrepreneurs (DEs) differ according to time and place. Nine issues were raised specifically throughout the interviews; these are included in Table 3, while other issues were brought up less frequently and with lesser significance. The following issues are prioritized in descending order of importance: inability to secure the funding needed under reasonable, realistic conditions and guidelines; failures and weaknesses in the face of unforeseen risks; inability to provide necessary advice and ongoing guidance; economic barriers and challenges; difficulties arising from intense pressure to compete locally, regionally, and internationally; inability to create and adopt a welcoming environment for entrepreneurs; inability to amend laws to keep up with swift changes; inability to manage various teams operating in Jordan.

**Table 3:** Major challenges and barriers that are facing digital startups entrepreneurs in Jordan are represented by frequencies and percentages. (Source: Author's own work).

Challenge	Frequency*	Percentage**
**Weakness in the funding required within fair, realistic conditions and criteria**	56	65.88 %
**Weaknesses and failures in the face of unexpected risks**	53	62.35 %
**Weakness in providing the necessary advice and continuous guidance**	50	58.82 %
**Economic barriers and challenges**	47	55.29 %
**Challenges of intense competitive pressures locally, regionally, and globally**	45	52.94 %
**Weakness Providing and adopting a friendly environment for entrepreneurs**	39	45.88 %
**Weakness in amending legislation and laws to keep pace with rapid changes**	31	36.47 %
**Weaknesses and obstacles in accessing different markets**	29	34.11 %
**Weakness in managing different teams**	21	24.70 %

*The frequency of each challenge/barrier is calculated for (n = 85) ** Percentage is calculated out (n = 85).

Similarities to the Jordanian situation described in the document can be seen when comparing DE in various nations, such as Africa. According to the research, African DE contributes little to the digital infrastructure, has trouble attracting venture funding, shows slow growth potential, and does not disrupt existing products and sectors. It also has limited prospects for international expansion. Furthermore, entrepreneurial learning presents difficulties for Jordanian and African DE, requiring regular modifications to strategies and methods [86], and [57]. [87]. These difficulties, which were two of the nine difficulties mentioned in the book, involve changes in team spirit and business model alterations. Interestingly, the remaining hazards on the list are more than tripled by the top five problems, indicating the need for a more thorough analysis in this chapter.

### 4.1 Challenge 1: weakness in the funding required within fair, realistic conditions and criteria

According to the survey, 65.88 % of the interviewees reported having trouble getting guaranteed pipeline access and insufficient money. At 65.88 %, the majority of respondents who were digital entrepreneurs agreed that there is a deficiency in both the application of fairness in the distribution of financial allocations to borrowers from digital entrepreneurs and the financial financing needed to start their entrepreneurial projects. Based on the firsthand experiences of the survey's target group, which is Jordanian entrepreneurs, this percentage was represented for all study industries. This could be because of the nation's inadequate financial resources. Due to its lack of wealth, as well as the fact that no clear laws, plans, or procedures have been adopted to assist business owners in establishing their ventures and putting them into action, the state's unemployment rate has decreased and its economic growth has increased.

Some digital firms might have modest finance, but others need more money to get off the ground and continue developing their products. The participants shared their viewpoints on the subject:

“*There is a common misconception that the capital for digital startups is just a laptop and the Internet. Unfortunately, this perspective is superficial*" ∼ (X).

“*Funding is necessary for digital startups to obtain software licenses, servers, domains, and advanced hardware, particularly for those utilizing AI and cloud computing. In contrast, non-digital startups may not incur all these expenses*” ∼ (Y).

“*The funding required varies depending on the scope of the idea and the necessary software and hardware. Additionally, it is essential to take into account the costs associated with marketing and operations*" ∼ (Z).

Early DEs encounter difficulties in comprehending the conditions for project finance, the actions that must be taken, and the assurances that must be obtained. Interviewees had a number of concerns during the process about the way qualifying projects are selected; they said that the procedure is opaque and does not meet requirements for integrity and transparency. In this instance, they also added:

“*Institutions base their funding decisions on the potential benefits they can gain, rather than personal attributes such as appearance or charm. This underscores their awareness of their own interests*” ∼ (W).

“*Some investors may request a stake in the company, which can lead to resentment among the founding team*” ∼ (F).

“*Institutions prioritize funding based on the potential benefits they can obtain, rather than personal characteristics like appearance or charm. They are fully aware of their own advantages*” ∼ (H).

“*Due to the pegging of the Jordanian dinar to the US dollar, applying for a bank loan during this period carries risks. This is because local interest rates are influenced by the procedures of the US Federal Bank, leading to higher interest rates locally*”∼ (T).

As a result, a lot of DEs like to finance their companies on their own, while some decide to take part in modest challenges that provide grants and prizes. Two respondents talked about their experiences:

“*I engage in challenges as a means to secure financial resources; otherwise, I would need to endure a longer wait to find new backers and investors*” ∼ (O).

“*Securing funding for startups presents a difficult choice where individuals must decide between two undesirable options*” ∼ (E).

These findings, which are based on the perspectives of the entrepreneurs who were questioned, are comparable to those of other earlier research, including [14,13], and [88]. However, there was some inconsistency between it and certain other studies, such as [20,89].

Following an interview, one of the middle-level managers expressed the following opinions:

*“The Ministry of Digital Economy and Entrepreneurship provides the necessary IT infrastructure for entrepreneurs to facilitate communication processes internally and externally and provides the necessary financial support and financing for the success of their businesses and facilitates procedures"∼* (D).

Another senior manager had his/her opinion as follows:

*“The Ministry of Digital Economy and Entrepreneurship frequently facilitates procedures with regard to the necessary licenses for start-ups and digital entrepreneurs and provides all sources related to business technology such as artificial intelligence, cloud computing, etc. to keep pace with the rapid technological* progress*"∼* (I).

The opinion of one of the directors was the following:

*“The financing provided by the Ministry of Digital Economy and Entrepreneurship is commensurate with the company's pioneering idea, the size of the startup and its operations, including necessary and required systems, devices, and programs needed*"∼ (J).

One of the biggest obstacles that entrepreneurs continue to confront is raising money for their startups. In order to get over the financial barriers they face, particularly in the research and development phases, they look into a variety of options [90]. DEs in Asian nations are also having financial difficulties, which has prompted them to use unusual strategies to deal with their restricted income flow [91].

### 4.2 Challenge 2: weaknesses and failures in the face of unexpected risks

The (n = 85) interviews revealed weaknesses and failures in the face of unforeseen dangers, as they accounted for 62.35 % of the total. DEs are always afraid about unanticipated dangers. At a rate of 62.35 %, the majority of respondents who identified as digital entrepreneurs acknowledged that they lacked the necessary tools from government agencies that support this industry, such as specialized courses or workshops, and that they were ill-prepared to handle unforeseen risks during and after the launch of their entrepreneurial projects. Based on the personal experiences of the survey's target group, which is Jordanian entrepreneurs, this percentage was represented for all study industries. This could be because of a lack of resources to develop and implement specialized risk management courses and reduce risks, both internal and external. It could also be because there aren't clear policies, strategies, or methods in place to assist entrepreneurs in implementing these programs when they start their projects. and put it into practice to lower risks and raise the likelihood that their initiatives will succeed in order to boost the state's economy and lower unemployment rates.

*“Entrepreneurship involves embracing risks, and that is precisely what we do"* ∼ (T).

*“Risks are ever-present in various aspects, encompassing technical challenges, market uncertainties, financial risks, and geopolitical instabilities in the region"* ∼ (B).

According to the interviewees, technological hazards are among the unexpected dangers. These could include unexpected product malfunctions, programming issues (errors and bugs), and hardware issues, as mentioned in the following excerpts:

*“I examined a website prior to meeting a client, but to my surprise, it was not functioning when I presented it during our discussion. It was an unforeseen and challenging situation, and I am still unsure about what went wrong at that moment"* ∼ (A).

*“I often find myself occupied with rectifying errors rather than focusing on the actual development processes"* ∼ (D).

*“Technical errors are bound to happen when dealing with programming and large files. Sometimes, I write over 50 lines of code in a day, and others write even more. Mistakes and unexpected issues can occur in such situations"* ∼ (H).

The findings presented above, which were derived from the perspectives of the entrepreneurs surveyed, are consistent with findings from other earlier studies, including [92,35]. On the other hand, there was some inconsistency between it and certain other studies, such as [25,47], and [49].

A director at the Ministry of Digital Economy and Entrepreneurship stated the following:

*“Any entrepreneurial idea within the scope of digital entrepreneurship, the element of risk in its application is present, but in different proportions commensurate with the size and type of the entrepreneurial idea presented in its chances of success*"∼ (V).

Another manager says:

*“The ministry provides specialized scientific courses in the field of risk management that digital entrepreneurs may face, such as various market risks, competitor risks, necessary financing risks, internal and external threats, logistical risks as well as geopolitical risks, etc.”* ∼ (C).

A director at the Ministry of Digital Economy and Entrepreneurship stated the following:

*“The Ministry works with digital entrepreneurs and helps them reduce and mitigate the risks that they may face while implementing their ideas, as well as providing the necessary support for the success of their entrepreneurial ideas to deal with the various risks smoothly, quickly, and with deliberate steps*"∼ (G).

DEs face issues with the IT infrastructure, which could prevent them from being able to make investments. In order to control these issues, startups work to enhance the digital infrastructure and seize excellent prospects for cooperation [16]. Many businesses face digital challenges that cause them to postpone product launches or seize early expansion opportunities [93,94], and [18].

### 4.3 Challenge 3: weakness in providing the necessary advice and continuous guidance

As shown in Table 3, the DEs rank the difficulty of providing insufficient direct advice and counseling as the third biggest challenge, accounting for 58.82 % of the challenges. Every DE is housed in an incubator that is either independent or connected to a university. Many of them did, however, voice concerns regarding the inadequate supervision. The majority of digital entrepreneurs who responded to the survey—58.82 % of them—confirmed that there is a glaring weakness in the way government organizations that support the digital entrepreneur sector reach out to them, as well as in the way they facilitate procedures and offer advice and guidance to them before and during the launch of their various entrepreneurial projects in several fields. Based on the personal experiences of the survey's target group, which is Jordanian entrepreneurs, this percentage was represented for all study industries. This could be because of a lack of ability to prepare and update the routine procedures, as well as to update the laws and programs required to facilitate the procedures and quickly obtain the necessary and sufficient support. It could also be because of a lack of ability to expedite the procedures in order to keep up with the rapid developments in a variety of fields. In addition to implementing clear policies, strategies, or methodologies to assist pioneering businesses in adopting such programs when entrepreneurs establish their projects and translate them on the ground to reduce risks and increase the chances of success of their projects to increase the state's economic growth and reduce unemployment rates.

The participants shared their experiences:

“*At first glance, the university appears to be promoting the entrepreneurial culture through entrepreneurship centers and incubators. However, upon closer examination, it becomes apparent that digital entrepreneurs are left to face the challenges on their own*" ∼ (M).

“*My incubator lacks a supervisor! … I'm not exaggerating, which is why I only go there when events are taking place*" ∼ (D).

During the interviews, the issue of supervisors lacking enough experience or competence was raised, which has an impact on DEs' performance and may divert their emphasis from product development to problem solving. The interviewees said:

“*Supervising incubators necessitates a diverse range of experiences, along with technical knowledge, as it embodies the essence of digital entrepreneurship*" ∼ (R).

“*The supervisor at the incubator in my university is a final-year student who lacks sufficient knowledge in many entrepreneurship topics and technical matters such as coding. Moreover, she is often preoccupied with her exams and graduation project*" ∼ (K).

“*In the past, I required technical assistance for my digital project, but unfortunately, I couldn't find the right specialist. Additionally, many supervisors in these incubators lack entrepreneurial experience or sufficient academic and practical expertise*" ∼ (M).

DEs often seek assistance from external sources, such as close friends, fellow entrepreneurs, experienced networks, and family members. While this may enhance their networking and communication skills, it can be time-consuming:

*“As a young entrepreneur, my main objective in participating in the incubator is to bridge the gaps in knowledge and technical skills. It would be challenging to accept the idea of not receiving assistance"* ∼ (S).

*“I dedicate a significant amount of time to seeking help and arranging meetings. If I invest this time in my product, I could achieve something remarkable"* ∼ (Z).

These findings, based on the opinions of the interviewed entrepreneurs, are consistent with earlier research [13,86,55], and [95]. While it was not completely compatible with other research such as [96,97], and [98].

The opinion of one of the directors at the Ministry of Digital Economy and Entrepreneurship was as follows:

*“The ministry has a qualified staff to provide advice, guidance, and advice to digital entrepreneurs, as well as reduce the obstacles and challenges that they may face before and during the start-up company"*∼ (Q).

Another manager says:

*“The ministry has the necessary expertise and qualifications technically, scientifically, and practically in terms of technical and theoretical knowledge regarding established companies and the requirements of their work and success*"∼ (L).

A director at the Ministry of Digital Economy and Entrepreneurship stated the following:

*“The Ministry is trying to work at its maximum capacity in serving digital entrepreneurs and overcoming challenges and obstacles as quickly as possible and working to solve them, as well as urging and attracting young energies with their digital entrepreneurial ideas and business incubators to bridge knowledge and technical gaps and work to adopt them*"∼ (N).

Given the rapid changes in the business world and the accelerated development of new technologies such as AI, the Internet of Things, and blockchain, it is critical to provide frontline advisory support to digital entrepreneurs and help them improve their abilities. Universities have an important role in developing the skills of entrepreneurs during the digital revolution [99].

### 4.4 Challenge 4: economic barriers and challenges

This challenge is related to outside variables, particularly the state of the economy. A little over half of the respondents—55.29 percent—think that the obstacles and difficulties they face on the financial front directly influence their digital enterprises and may even create new ones. The majority of respondents, who were digital entrepreneurs, or 55.29 % of the sample, acknowledged that they face definite financial difficulties and roadblocks both before and after launching their various business ventures. They also acknowledged that government organizations that support this industry are underequipped to handle these issues. Based on the personal experiences of the survey's target group, which is Jordanian entrepreneurs, this percentage was represented for all study industries. This could be the result of Jordan's limited capacity to support and embrace entrepreneurs through the provision of support programs. In addition to overcoming barriers to receiving sufficient financial and moral support for them by speeding up economic measures that assist them and providing all the resources needed for the success of their innovative ideas and putting them into practice to keep up with the quick developments in various spheres of life, there should also be clear policies, strategies, or methodologies in place to assist entrepreneurs in adopting such supportive economic programs in order to lower the risks of their failure and increase the likelihood that their projects will succeed in order to boost the state's economy and lower unemployment rates.

Some interviewees provided insights:

“*I meticulously review the price offer on multiple occasions before presenting it to the customer, as I am fully aware that price holds significant importance for a considerable portion of our customer base*." ∼ (R).

*“The influence of the market size in Jordan contrasts with the impact of the economic situation on Des*” ∼ (S).

*“The economic dimension extends beyond the local level and has repercussions on a global level*” ∼ (Z).

Customers' purchasing power is being severely curtailed by the dire economic conditions in several nations, especially the Middle East, which is forcing many of them to reevaluate their basic demands. Because they require more work during development and integration than more basic digital services, digital products that use AI and cutting-edge technology are more expensive. The cost of the product reflects this:

“*Examine the pricing of AI-driven products. Our target audience is specific, and we acknowledge that not everyone may fully comprehend the pricing structure of AI products*" ∼ (A).

“*The operational expenses associated with advanced technology create challenges for DEs themselves and these challenges are ultimately passed on to customers*" ∼ (T).

The perspectives of the entrepreneurs who were interviewed and the results as displayed above are compared with those of other earlier research, including [63,1,100], and [101]. On the other hand, there was some inconsistency between it and certain other studies, such as [91,102].

A director at the Ministry of Digital Economy and Entrepreneurship stated the following:

*“From the point of view of the ministry, as well as the digital entrepreneurs, the economy based on their commercial activities is not confined locally within a specific geographical area*"∼ (K).

Another senior manager says:

*“From the Ministry's point of view, technological and operational costs are among the most important challenges and economic obstacles for digital entrepreneurs*"∼ (B).

The economy and digital entrepreneurship are intertwined. Economic development depends heavily on entrepreneurial enterprises (DEs), and DEs are impacted by changes in the economy [100]. confirmed that developing enterprises are greatly impacted by economic situations. Furthermore, a diminished function of business incubators in promoting startups was noted. There is an emphasis on coaching DEs' financial literacy in order to assist them overcome future issues, given the importance of understanding the financial obstacles faced by entrepreneurial enterprises, particularly economic situations [103].

### 4.5 Challenge 5: challenges of intense competitive pressures locally, regionally, and globally

All of the interviewees agreed that working in the digital space exposes them to different kinds of competition. This competition involves 52.94 % of DEs from other nations in addition to domestic competitors. Even with their startup expertise, many startups struggle to compete against more established companies both locally and globally. At 52.94 %, the majority of respondents' perceptions of digital entrepreneurs were centered on the significant obstacles and competitive pressures they face on a local, regional, and worldwide scale. This necessitates the use of all capabilities by government or private agencies that support programs that assist digital entrepreneurs in launching their entrepreneurial projects and ideas to provide high-quality and unique products or services in order to gain distinct competitive advantages and increase their chances of success in competition with other local or foreign entrepreneurial projects. This percentage was reflected in all industries covered in the survey, based on the various viewpoints and personal experiences of the target group of Jordanian entrepreneurs. As a result, it is necessary to overcome all obstacles and provide all of the resources and sources required to obtain adequate economic and moral support for them by accelerating economic measures supporting them and providing all of the necessary sources for the success of their creative ideas and their implementation on the ground in order to keep up with the rapid developments in the various fields of life. Furthermore, clear policies, strategies, or methodologies should be adopted to assist entrepreneurs in implementing such supportive economic programs in order to reduce the risks of failure and increase the chances of success of their projects, thereby increasing the country's economic growth and lowering unemployment rates.

The interviewees shared their perspectives:

“*The presence of prominent digital competitors leads to more than half of new DEs abandoning their projects within the first year*" ∼ (K).

“*External competitors are an indispensable aspect of the competitive landscape*" ∼ (Z).

“*It is challenging for me to compete with major website/app builders globally who leverage a multitude of ready-made templates and sometimes charge customers exclusively for hosting services. In contrast, I dedicate hours to programming, customization, and design*" ∼ (D).

Digital entrepreneurship involves a constant adaptation of the business strategy to meet the ever-changing market and client demands. As a result, a solution that works well in one country may not be suitable in another, posing new issues for DEs.

“*Merely integrating technology into your startup is insufficient as technology continues to advance*" ∼ (H).

“*Employing advanced technology can offer a competitive edge, but it is not sufficient when faced with competitors"* ∼ (M).

“*Consider the larger companies … They consistently roll out updates, so it's challenging for smaller companies to keep pace*!" ∼ (S).

These findings, based on the opinions of the interviewed entrepreneurs, are consistent with earlier research [104,105], and [106]. While it was not completely compatible with several other investigations, such as [96,97].

A director at the Ministry of Digital Economy and Entrepreneurship stated the following:

*“There is a challenges of intense competition in the environment of digital entrepreneurs and startups, and often more than half of the entrepreneurs are unable to proceed with their entrepreneurial projects, especially in the first three years of their launch*"∼ (S).

Another senior manager says:

*“From the point of view of an experienced manager in serving digital entrepreneurs and startups, intense competition these days is not limited to providing technology and its various uses only to entrepreneurs, but rather to the quality of distinguished service provided to customers*"∼ (U).

A director at the Ministry of Digital Economy and Entrepreneurship stated the following:

*“Most of the large-scale companies working in digital entrepreneurship and startups are modernizing their operational, administrative, and logistical systems and adopting the latest technological technologies to keep pace with the rapid developments to serve customers in a more distinctive way regionally and globally than companies with limited resources and capabilities in their scope of work and capabilities locally*"∼ (F).

While competitiveness is a key difficulty for DEs, other challenges include obtaining funds, economic considerations, and dealing with numerous administrative issues within their teams. Human resource management leadership is critical to a startup's success. Overcoming these obstacles is critical to the sustainability and growth of DEs [102].

Additionally, DEs face additional problems relating to their staff and talent. These problems include sourcing internationally skilled personnel, such as software engineers, who specialize in high-demand specialist sectors like the Internet of Things, Fintech, and algorithms [86].

Challenge 6: Weakness providing and adopting a friendly environment and sustainability for entrepreneurs.

Digital entrepreneurship has a bright future, thanks to the increased reliance on digital platforms during the COVID-19 epidemic. DEs are aggressively adopting technology into their projects and using globalization to broaden their reach [25]. However, early-stage DEs in developing countries face various hurdles, including insufficient finance, challenging economic conditions, a failure to provide and adopt a hospitable environment for entrepreneurs, fierce competition, and unforeseen dangers, accounting for 45.88 %. As a result, DEs are continuously looking for ways to reduce these risks and raise the likelihood that their project will succeed. The opinions of less than half of the targeted respondents from digital entrepreneurs, at a rate of 45.88 %, were that government or private agencies that support programs for adopting digital entrepreneurs in launching their projects and green entrepreneurial ideas to provide products or services of high quality and uniqueness, do not adopt programs or provide them with sources for them to be friendly and green to the environment. In today's business world, we must provide all technologies and tools that take into account the environment and reduce the negative effects of its operational processes through the use of production requirements that can be naturally analyzed over time, and preserve the environment and its sustainability by raising awareness of digital entrepreneurs in Jordan in order to increase its chances of success and competition with other pioneering local or foreign environments. This percentage was reflected for all industries covered in the survey, based on the diverse viewpoints and personal experiences of the target group of Jordanian entrepreneurs. As a result, it is necessary to overcome all obstacles and provide all of the necessary resources and resources so that they can compete with other projects in order to obtain adequate economic and moral support by accelerating the economic measures supporting them and providing all of the necessary sources for the success of their creative ideas and their application on the ground. To keep up with rapid changes in numerous spheres of life, in addition to implementing clear green policies, strategies, or methodologies that consider and retain the support of green entrepreneurs in adopting such programs.

The interviewees shared their perspectives:

“*We offer all necessary resources so that we can environmentally be friendly so that we can compete with other projects to obtain adequate support for our startup economically and morally by accelerating the economic measures supporting us and providing all the necessary sources for the success of our creative ideas and our applications on the ground for customers*" ∼ (K).

A director at the Ministry of Digital Economy and Entrepreneurship stated the following:

*“The Ministry provides adequate support of all kinds, whether material or moral green, as well as facilitation and speed in procedures for startups and digital entrepreneurs in providing everything necessary for the success of their entrepreneurial projects in a short time and become more sustainable* "∼ (A).

A director at the Ministry of Digital Economy and Entrepreneurship stated the following:

*“The Ministry provides sufficient support of all kinds to all emerging companies and digital entrepreneurs in providing everything necessary to overcome obstacles to the success of their entrepreneurial projects and facilitate their access to different markets"*∼ (W).

Another senior manager says:

*“The strategy and methodology that the Ministry relies on to overcome all the challenges that emerging companies and digital entrepreneurs may face are harnessing all resources, capabilities, and agreements concluded with other friendly and brotherly countries and various communication networks in order to make their entrepreneurial projects a success and facilitate their access to different markets by providing products or services distinctive for clients*" ∼ (J).

These findings, based on the opinions of the interviewed entrepreneurs, are consistent with earlier research [86,24], and [15]. While it was not completely consistent with several other studies, such as [107,37].

A director at the Ministry of Digital Economy and Entrepreneurship stated the following:

*“The Ministry has the ability to organize its business and activities in order to make startups and digital entrepreneurs succeed in applying their entrepreneurial ideas and translating them into reality, in addition to increasing their chances of success in the highly competitive business environment and dynamic markets*"∼ (U).

A director at the Ministry of Digital Economy and Entrepreneurship stated the following:

*“The strategy and methodology that the ministry relies on is joint work through specialized teams with experience and knowledge in providing the necessary advice and support required for startups and digital entrepreneurs in order to raise their capabilities and chances of success in a volatile business environment and markets by building participatory and integration*"∼ (P).

Another senior manager says:

*“The Ministry has the ability and competence to manage different teams within various activities and specializations in building joint work, local, regional, or international entities or institutions to provide the necessary and required advice and support for startups and digital entrepreneurs in order to raise their capabilities and chances of success in a volatile business environment and markets*"∼ (L).

The analysis also revealed that some entrepreneurs are opting to self-employment to avoid unemployment, potentially reducing pressure on both public and private companies. However, early-stage DEs face major challenges in obtaining funding for their projects and getting venture capital. They prefer easy and transparent financial options. Unfortunately, many investors set onerous requirements on emerging entrepreneurs, limiting their growth and development.

Arabic countries, like Jordan, continue to lack the required support and awareness for digital entrepreneurship, entrepreneurship, and innovation in general [108], and [109]. As a result, this study stresses the importance of promoting DE, as it can help to reduce unemployment and create new prospects for economic and social development. Providing sufficient assistance and counsel to entrepreneurs is critical in this regard. The quick expansion of DE operations can lead to project development and new possibilities, resulting in more job opportunities and lower unemployment rates. Entrepreneurs can apply their digital skills to many areas of the Jordanian business landscape, increasing the competitive advantage of multiple stakeholders in terms of innovation and sustainability. It is worth noting that this study will be broadened to produce additional insights and conclusions that reflect the distinct Arab context or regional landscape of digital entrepreneurship.

Furthermore, incubators play a critical and underappreciated role in teaching DEs risk management and evaluation. DEs should learn how to create backup plans and assess the possibility and impact of hazards.

In summary, and in light of the aforementioned findings, we suggest the following key recommendations to those in charge of formulating government policies and initiatives:

➢ Boost the system's level of convenience to expedite the processes and regulations enabling digital businesses to obtain the necessary money and loans quickly and effortlessly;
➢ Examine the laws again and attempt to adjust guidelines and directives to accommodate the rapid changes in the world;
➢ To provide digital entrepreneurs with specialized scientific courses in risk management, the Ministry of Digital Economy and Entrepreneurship should expand the number of its training programs. These courses should cover various risks that digital entrepreneurs may encounter, including market risks, competitor risks, risks related to necessary financing, internal and external threats, logistical risks, and geopolitical risks.
➢ Raising awareness of digital entrepreneurs is possible thanks to the Ministry of Digital Economy and Entrepreneurship, which is doing everything it can to support these business owners by identifying and resolving problems as soon as they arise. In addition, they inspire and draw in young people with their digital business concepts and incubators, pushing them to close knowledge and technological gaps and strive toward adoption.
➢ Offer complete financial and non-financial support to digital entrepreneurs so that the economy built on their business ventures is not limited to a certain region.

The Ministry of Digital Economy and Entrepreneurship employs modern and flexible strategies and techniques to surmount any obstacles that may arise for nascent enterprises and digital entrepreneurs. These include leveraging all available resources, capacities, and agreements reached with friendly and neighboring nations, as well as diverse communication channels, to ensure the success of their entrepreneurial endeavors and to ease their entry into new markets by offering unique products or services to customers.

## 5 Conclusion

People are starting to engage in digital entrepreneurship (DE) because of the COVID-19 epidemic, which has caused a boom in digital transformation, and Jordan's high unemployment rate. But when they go out on this adventure, they run across a number of difficulties. Research using a qualitative approach is being done to investigate these issues.

Early DEs are actively looking for funding options that are transparent and feasible. In an attempt to improve their market presence and obtain a competitive advantage, a large number of them are investing in the development of their digital platforms. Obtaining sufficient funds is essential to this procedure. The emergence and expansion of digital companies relieves pressure on employment authorities while also lowering unemployment rates. Furthermore, it creates opportunities for foreign investment in the regional digital economy, which eventually improves Jordan's digital and entrepreneurial scene. In order to improve investment and finance alternatives for early DEs, this report proposes additional funding sources, streamlined processes, and award opportunities. It also suggests that centers and incubators for entrepreneurship provide all-encompassing advice, one-on-one coaching, and work with outside specialists. It is crucial to update the laws and rules pertaining to business registration in the digital age, with an emphasis on creating and managing an environment that encourages entrepreneurship.

While this study focuses especially on Jordan, it is possible to apply these conclusions to other developing countries experiencing similar challenges, particularly those coping with high unemployment rates. Furthermore, based on earlier studies and analyses, there are still chances to investigate the motivations and interpersonal and intrapersonal issues faced by DEs, with a particular focus on developing a more comprehensive knowledge of their unique consequences.

### 5.1 Theoretical and practical implications

This study expands upon prior research that evaluated the key challenges experienced by digital entrepreneurs, particularly in developing nations. This study offers information that can reduce costs, boost efficacy and efficiency, and improve overall performance; therefore, executives and decision-makers must take it seriously [43], and [39]. By focusing on nine categories of obstacles—including institutional, technological, and local factors—this study expands the field of entrepreneurial research. It expands our knowledge of the relationship between context and entrepreneurship by illuminating how digital entrepreneurs maneuver their surroundings and view context as either an asset (opportunities) or a liability (challenges) [104,110,105], and [106].

Based on the study's findings, a number of significant managerial and practical ramifications have been identified to promote digital entrepreneurship and assist nascent enterprises in overcoming the major roadblocks and difficulties they may face before to or during their debut. First and foremost, developing a communication and information technology infrastructure can help streamline and expedite processes in order to work toward sustainable financing of innovative initiatives and start-ups. The advancements in banking and digital services, facilitated by broadband internet, have created opportunities for digital businesses to access internet banking services [88], and [111]. The popularity of mPesa in Kenya serves as one example of this. The expansion of internet-enabled SMEs in India has also been facilitated by government initiatives that encourage the penetration and adoption of ICTs and the internet [34]. Applying what has been learned from these experiences to Cameroon could improve market access in areas where logistical challenges hamper physical market access; however, online platforms can facilitate commercial activities, reduce research expenses, and strengthen the links between the local technological context and institutional setting.

Second, the study emphasizes the importance of specialized training in acquiring direct and simplified financing, ensuring its sustainability and efficiency, and advising and supporting businesses in technical areas from both the public and private sector. Addressing numerous dangers and modernizing information and communication technology incubators, such as Active Spaces [95], are critical measures. Along with making investment money more accessible, addressing financial limitations and revising laws and regulations are also crucial [96]. Additionally, IT departments can facilitate relationships with clients and outside logistics suppliers [107], as well as providing access to technology alliances and networks for business development while boosting human capital and entrepreneurial awareness [26]. By taking these steps, we can make sure that the technical environment works to the benefit of digital entrepreneurs rather than against them.

This study makes a significant contribution, although there are certain drawbacks that came up during execution. First, this study concentrated on only digital entrepreneurs in some specific and limited number of start-ups sectors in Jordan as a developing country specifically, as the target group was only from the State of Jordan. Nevertheless, the current study's limitations limit how broadly the findings may be applied. Additionally, the study's findings might not be applicable to digital entrepreneurs in other parts of the globe or in nations with different cultures, thought processes, educational backgrounds, legal frameworks, etc. As a result, scholars can take advantage of this and broaden the study's scope to encompass several additional nations and consider these contexts either as a whole or in parts. Second, it was challenging to generalize the study's findings since only in-depth interviews with managers in the Ministry of Digital Economy and Entrepreneurship operating in Jordan or digital entrepreneurs were used as the methodology. To raise the degree of credibility of the findings, researchers are therefore encouraged to undertake experimental and longitudinal designs in the future. The small group of digital entrepreneurs that attended, along with decision-makers from ministries and other public and private organizations (banks, etc.), had to do with supporting processes and implementing the concepts of digital entrepreneurs to make them a reality.

Prior to this research, there was a dearth of understanding about the major roadblocks and hurdles that could stymie the advancement of digital entrepreneurs and start-ups. As a result, there is a need to broaden the scope, focus more on sustainable digital entrepreneurship, include more developing countries, and develop a more precise perspective in order to make informed decisions and take the necessary steps to address and mitigate the obstacles and challenges that digital entrepreneurs face.

Additionally, we urge academics and researchers to concentrate more of their future work on examining each startup or entrepreneur sector alone rather than examining all of them collectively in order to compare and contrast them and highlight any discrepancies using additional variables. This can be accomplished through encouraging organizational adaptability and streamlining processes. Therefore, it is highly advised that more research be done on a variety of start-ups in the Arab world, utilizing longitudinal studies as opposed to only cross-sectional ones like this one. Additionally, we propose adopting and implementing mixed research technique, which incorporates quantitative via surveys, and qualitative via in-depth interviews to get more dependable and accurate conclusions. The study's conclusions set the stage for the creation of assessment instruments that will gauge donors' and entrepreneurs' degree of engagement as well as the potency of resilience-building techniques. The conceptual framework used in this study highlights the resilience of small and medium-sized firms (SMEs) and the crucial role that entrepreneurs play in the context of digital sustainability by bringing together several management and resilience research viewpoints.

## Data availability statement

Data will be made available on request by the authors.

## Funding statement

This study is not funded by any entity.

## CRediT authorship contribution statement

**Moh'd Anwer AL-Shboul:** Conceptualization, Formal analysis, Investigation, Methodology, Resources, Supervision, Validation, Visualization, Writing – original draft, Writing – review & editing.

## Declaration of competing interest

I hereby declare that the disclosed information is correct and that no other situation of real, potential or apparent conflict of interest is known to me. I undertake to inform you of any change in these circumstances, including if an issue arises that is related to my paper.

We wish to confirm that there are no known conflicts of interest associated with this publication and there has been no significant financial support for this work that could have influenced our outcome.

No funding was received for this work.
